This article has been retracted.

# Risk Factors of Periodontal Disease: Review of the Literature

**DOI:** 10.1155/2014/182513

**Published:** 2014-05-20

**Authors:** Yousef A. AlJehani

**Affiliations:** Dental Health Department, College of Applied Medical Sciences, King Saud University, P.O. Box 10219, Riyadh 11433, Saudi Arabia

## Abstract

*Objectives*. This paper aims to review the evidence on the potential roles of modifiable and nonmodifiable risk factors associated with periodontal disease. *Data*. Original articles that reported on the risk factors for periodontal disease were included. *Sources*. MEDLINE (1980 to Jan 2014), PubMed (using medical subject headings), and Google Scholar were searched using the following terms in different combinations: “periodontal disease,” “periodontitis,” “risk factors,” and “causal.” This was supplemented by hand-searching in peer-reviewed journals and cross-referenced with the articles accessed. *Conclusions*. It is important to understand the etiological factors and the pathogenesis of periodontal disease to recognize and appreciate the associated risk factors. As periodontal disease is multifactorial, effective disease management requires a clear understanding of all the associated risk factors.

## 1. Introduction

Periodontitis is one of the most ubiquitous diseases and is characterized by the destruction of connective tissue and dental bone support following an inflammatory host response secondary to infection by periodontal bacteria [1, 2]. Severe periodontitis, which may result in tooth loss, is found in 5–20% of most adult populations worldwide [3–5]. Children and adolescents can have any of the several forms of periodontitis such as aggressive periodontitis, chronic periodontitis, and periodontitis as a manifestation of systemic diseases [6–8].

It is now generally agreed that almost all forms of periodontal disease occur as a result of mixed microbial infections within which specific groups of pathogenic bacteria coexist [9–11]. Evidence is reviewed on the potential roles of modifiable and nonmodifiable risk factors associated with periodontal disease. An understanding of risk factors is essential for clinical practice.

### 1.1. Search Strategy

MEDLINE (1980 to Jan 2014), PubMed (using medical subject headings), and Google Scholar were searched using the following terms in different combinations: “periodontal disease,” “periodontitis,” “risk factors,” and “causal.” This was supplemented by hand-searching in peer-reviewed journals and cross-referenced with the articles accessed.

## 2. Risk Factors of Periodontal Disease

### 2.1. Modifiable Risk Factors

#### 2.1.1. Microorganisms and Periodontal Disease

The oral bacterial microbiome includes over 700 different phylotypes, with approximately 400 species found in subgingival plaque [12, 13]. The subgingival microflora in periodontitis can harbor hundreds of bacterial species but only a small number has been associated with the progression of disease and considered etiologically important. Subgingival plaque from deepened periodontal pockets is dominated by gram-negative anaerobic rods and spirochetes [14, 15]. Strong evidence has implicated* Porphyromonas gingivalis* [16] and* Aggregatibacter actinomycetemcomitans* [17, 18] to the pathogenesis of adult periodontitis. In addition,* Bacteroides forsythus* [19],* Prevotella intermedia* [18],* Peptostreptococcus micros* [20], and* Fusobacterium nucleatum* [21] have been strongly linked with the progression of adult periodontitis.

#### 2.1.2. Tobacco Smoking

There is accumulating evidence for a higher level of periodontal disease among smokers [22, 23]. Tobacco smoking exerts a substantial destructive effect on the periodontal tissues and increases the rate of periodontal disease progression [24]. Risk factors including tobacco smoking modify the host response to the challenge of bacteria in microbial dental plaque [25, 26]. Smokers with periodontal disease seem to show less signs of clinical inflammation and gingival bleeding compared to nonsmokers [27]. That could be explained by the fact that nicotine exerts local vasoconstriction, reducing blood flow, edema, and clinical signs of inflammation [28]. Nicotine acetylcholine receptor has been found to play an important role in the development of nicotine related periodontitis [29].

#### 2.1.3. Diabetes Mellitus

One of the important oral signs of diabetes is gingivitis and periodontitis. Patients with undiagnosed or poorly controlled diabetes mellitus type 1 or type 2 are at higher risk for periodontal disease. There are many studies that demonstrate an association between diabetes and an increased susceptibility to oral infections including periodontal disease [30–34]. Periodontitis also progresses more rapidly in poorly controlled diabetics [35], and early age of onset of the disease is seen as a risk factor for more severe diseases [36]. Conversely, most well-controlled diabetic patients can maintain periodontal health and will respond favorably to periodontal therapy [37].

Despite discrepancy regarding this issue in the scientific literature, it seems that the effect of glycemic control is related to the mode of periodontal therapy [38]. Many studies addressed the effect of periodontal treatment on glycemic control of diabetes patients [39–46].

#### 2.1.4. Cardiovascular Disease

The biological plausibility of the association between periodontal diseases and cardiovascular diseases is well studied and it includes some of the following possible mechanisms: high concentrations of cholesterol and the action of oral bacteria in the process of atherosclerosis or the participation of acute-phase proteins that may increase in chronic periodontitis [47, 48]. Several biological mechanisms have been proposed to explain the relationship between periodontal diseases and cardiovascular diseases. Therefore, periodontitis can probably elicit a systemic inflammatory response and it deserves more attention [49].

Periodontal disease is capable of predisposing to vascular disease due to the rich source of subgingival microbial species and host's response. Furthermore, we must be aware that these diseases share many risk factors and there are evident similarities to the basic pathogenic mechanisms [50].

Periodontitis is associated with the increase in the level of C-reactive protein and fibrinogen, irrespective of coronary diseases. Furthermore, there is evidence that suggests that the increase in the levels of systemic markers of inflammation, such as the C-reactive protein (CRP) and interleukin-6 (IL-6), is associated with cardiovascular diseases [51].

Bacteremia from periodontitis and dental disease is known to be the primary cause of infective endocarditis [52]. In particular, patients who have undergone heart valve surgery have a significant risk of life-threatening infective endocarditis. Epidemiological and microbiological studies have lent credence to the concept that periodontal disease may be a separate risk factor for cardiovascular disease, cerebrovascular disease [53], and preterm delivery of low birth weight infants [54].

Wu et al. [55] have shown that periodontal disease is another putative and independent risk factor for cerebrovascular disease, particularly for ischemic stroke. Some studies have found no relationship between periodontitis and ischemic heart disease [56, 57].

#### 2.1.5. Drug-Induced Disorders

Some medications significantly decrease salivary flow. These include antihypertensives, narcotic analgesics, some tranquilizers and sedatives, antihistamines, and antimetabolites. Other drugs, particularly those in liquid or chewable form that contain added sugar, alter the pH and composition of plaque, making it more able to adhere to tooth surfaces [58].

Drugs can be a contributing factor in periodontal diseases. Drugs such as anticonvulsants, calcium channel blocking agents, and cyclosporine may induce gingival overgrowth [59].

#### 2.1.6. Stress

Patients with inadequate stress behavior strategies (defensive coping) are at greater risk for severe periodontal disease [60–65]. Stress is associated with poor oral hygiene, increased glucocorticoid secretion that can depress immune function, increased insulin resistance, and potentially increased risk of periodontitis [66]. Men who reported being angry on a daily basis had a 43% higher risk of developing periodontitis compared with men who reported being angry seldom [66]. Studies have found some periodontal disease indicators such as tooth loss and gingival bleeding to be associated with work stress [66, 67] and financial strains [68].

#### 2.1.7. Obesity

Obesity has been reported to be an important risk factor for periodontal disease [69, 70]. Several explanations for the association between obesity and periodontal disease [71–73] in younger adults have been provided. Younger people may have different dietary patterns than older study participants. Research in dietary trends in adolescent's ages from 11 to 18 reveals a significant decrease in raw fruit and nonpotato vegetables, which are sources of vitamin C. In addition, adolescents have decreased their calcium intake and increased their intake of soft drinks and noncitrus juices. This is important to oral health because low dietary intake of calcium and vitamin C has been associated with periodontal disease [74]. People who consume less than the recommended dietary allowance (RDA) for calcium and vitamin C have slightly higher rates of periodontal disease [74].

### 2.2. Nonmodifiable Risk Factors

#### 2.2.1. Osteoporosis

Many of the studies conducted to date suggest there is a relationship between skeletal osteoporosis and bone loss [75–80] to the extent that postmenopausal osteoporosis may result in dental osteopenia involving the jaws, and particularly the mandible [81]. Osteoporosis was significantly associated with severe alveolar crestal bone loss and the prevalence of periodontitis cases in postmenopausal women [82]. A review of the relationship between osteopenia, oral bone loss, and periodontal disease [83, 84] concluded that osteopenia does play a role in the expression of periodontal disease. The review indicated a direct association between skeletal and mandibular osteopenia and loss of alveolar crestal height and tooth loss in postmenopausal women. Taguchi et al. [85] have stressed that it is important to distinguish among osteopenia, which has been defined in general terms as a decrease in normal mineralized bone, postmenopausal osteoporosis, which is a disease caused by the cessation of estrogen production and characterized by spinal fractures that occur between the ages of 50 and 70 years, and osteoporosis, which affects an older population and results in proximal femur fractures [86]. Periodontitis and osteopenia may have common etiological agents that may either directly influence or modulate both disease processes [87].

#### 2.2.2. Hematological Disorders

Hemorrhagic gingival overgrowth with or without necrosis is a common early manifestation of acute leukemia [88]. Patients with chronic leukemia may experience similar but less severe periodontal changes. Chemotherapy or therapy associated with bone marrow transplantation may also adversely affect the gingival health [89, 90].

#### 2.2.3. Host Response

Chronic periodontitis involves complex interactions between microbial factors and susceptible hosts [91, 92]. The bacterial components such as lipopolysaccharides and cytokines activate the macrophages to produce cytokines such as interleukin (IL)-1 and tumor necrosis factor (TNF) [39, 93]. These cytokines activate the fibroblasts that reside in the periodontal tissues to the matrix metalloproteinases (MMPs), a plasminogen activator, which can activate plasmin. Plasmin, in turn, can activate some other types of latent MMPs, while tissue inhibitors of metalloproteinases (TIMPs) can inactivate the active MMPs [94]. Among susceptible individuals, the prolonged and excessive bacterial promotions of the MMPs induce the enhanced degradation of collagen, which is a primary component of the periodontal matrix. MMP-8 and -9 are released from the polymorphonuclear leukocytes (PMN) and are responsible for a substantial part of the destruction caused by the host response. MMP-13 also facilitates bone resorption by degrading the collagenous matrix of the bone after the bone is demineralized by osteoclasts [95]. Marcaccini et al. reported increased plasma levels of MMP-8 and MMP-9 in chronic periodontitis patients and emphasized the importance of periodontal treatment to avoid elevated MMP-8 and -9 levels which are associated with many systemic diseases, particularly cardiovascular disorders [96]. A recent review on the modifiable risk factors concluded that smoking and excess caloric intake contribute to increases in systemic markers of inflammation and can modify gene regulation through a variety of biologic mechanisms [97].

#### 2.2.4. Female Hormonal Alterations

Hormonal fluctuations in the female patient may alter the status of periodontal health [98]. Such changes may occur during puberty, the menstrual cycle, pregnancy, or menopause. Changes may also be associated with the use of oral contraceptives. The most pronounced periodontal changes occur during pregnancy, as a significant proportion of pregnant women suffer from pregnancy gingivitis. Women on hormonal replacement therapy (HRT) and oral contraceptives experience increased gingival inflammation [81, 99]. With oral contraceptives, this increase in gingival inflammation is mainly related to the duration of use as it has been suggested that prolonged use of oral contraceptives may detrimentally affect the periodontium.

#### 2.2.5. Pregnancy

Offenbacher et al. [92] found significantly more periodontal attachment loss among mothers of PLBW infants compared with mothers of normal-term infants.

Similarly, several other studies have suggested an adverse influence of periodontal disease on the course of pregnancy [100–103]. It has been suggested that periodontal disease may increase the risk of having preterm low birth weight (PLBW) infants [104, 105]. This outcome is thought to be the effect of biologic mediators of inflammatory processes such as prostaglandins E2 and TNF. The common bacterial product lipopolysaccharide also may have a triggering role in adverse change of the course of pregnancy.

## 3. Risk Characteristics

### 3.1. Age

Several studies show that the prevalence and severity of periodontal disease increase with age [87, 106–112]. Papapanou et al. demonstrated that the mean annual rate of bone loss among the initially 70-year-old subjects was 0.28 mm compared to 0.07 on the 25-year-old individuals [112]. The increased severity of periodontal disease and bone loss with age is probably related to the length of time, where the periodontal tissues have been exposed to bacterial plaque, and is considered to reflect individual's cumulative oral history [113]. More studies carried out in some of the developed countries show changing patterns of periodontal disease progression. These studies have shown that advanced periodontal destruction and bone loss are seldom seen in individuals under the age of 40 [109, 114]. A similar finding has been observed even in the elderly population. Studies among the elderly have shown that advanced periodontal disease affects only a small fraction of this age group [108, 114]. However, among those with advanced disease, further breakdown does occur with increasing age.

### 3.2. Sex

Numerous studies reported higher periodontal destruction among males compared to the female population [87, 115–118]. The reasons for these sex differences are not clear, but they are thought to be related to the ignorance of oral hygiene, which is usually observed among males [118, 119]. However, the relationship observed between sex and the disease is not apparent and is not considered as strong and consistent. Thus, sex may be a demographic factor, which may interfere with the effects of other factors and it must be controlled for investigating the disease.

### 3.3. Socioeconomic Status (SES)

The possible relationship between periodontal disease and socioeconomic status was found in several studies [108, 110, 120–122]. Gingival condition is clearly related to lower SES, but the relationship between SES and periodontitis is less direct. It can be certain that gingival health is better among individuals with higher education and with more secure income. SES is a modifiable factor and it can be examined in multivariate models for the disease.

### 3.4. Education and Race

Periodontal disease has a reciprocal relationship with educational level. The higher the educational level, the lower the periodontal diseases (Department of Health Education and Welfare, 1966). Several studies involving different racial populations have found some difference in the expression of periodontal disease [108]. Once again, race is not a modifiable factor, and some discrepancies in disease expressions may be explained by the differences in other risk factors between populations.

### 3.5. Genetic Considerations

Studies show genetic risk factors associated with periodontitis [123–129]. McDevitt et al. demonstrate that the composite IL-1 genotype is significantly associated with the severity of adult periodontitis. They also confirmed that both IL-1 genotyping and smoking history provide objective risk factors for periodontal disease in a private practice environment [130]. Currently, there are two major forms of periodontitis-chronic and aggressive periodontitis [6]. Risk for periodontitis is not shared equally by the population. It is clear that periodontitis severely affects a high-risk group representing around 10–15% of the population, in whom the disease quickly progresses from chronic gingivitis to destructive periodontitis [131]. This differential risk for periodontitis is consistent with heritable elements of susceptibility, but direct evidence for a differential genetic contribution to periodontitis comes from several sources.

Many works of the literature report familial aggregation of periodontal diseases, but due to different terminology, classification systems, and lack of standardized methods of clinical examination, it is difficult to compare reports directly. Although periodontal disease nosology has changed many times over the timeframe of these reports, most familial reports for periodontitis are for early-onset forms now called aggressive periodontitis [132–139]. Reports of the familial nature of chronic forms of periodontitis are less frequent, although German studies of the familial nature of chronic forms of periodontitis from the early 20th century have been reviewed by [140]. This aggregation within families strongly suggests a genetic predisposition. It must be borne in mind that familial patterns may reflect exposure to common environmental factors within these families. Thus, it is important to consider the shared environmental and behavioral risk factors in any family. These would include education, socioeconomic grouping, oral hygiene, possible transmission of bacteria, incidence of chronic diseases such as diabetes, and environmental features, such as passive smoking and sanitation. Some of these factors, such as lifestyle, behavior, and education, may be under genetic control and may influence the standards of oral hygiene. The complex interactions between genes and the environment must also be considered in the evaluation of familial risk for the periodontal diseases.

In chronic periodontitis, the phenotype or disease characteristics do not present significantly until the third decade of life, whereas, in the aggressive forms of periodontal disease, the presentation can occur in the first, second, third, and fourth decades. This variability in presentation of significant signs of disease makes diagnosis difficult, not only in declaring if a patient suffers from the disease but also in detecting patients who do not suffer from the disease and differentiating between adult and aggressive forms of periodontitis. The problems associated with the clinical differentiation of periodontal disease are not uncommon in medical genetics, since similar problems arise in the study of other delayed-onset hereditary traits [133].

### 3.6. C-Reactive Protein

Cholesterol has long been known to play a crucial role in predicting risk for heart attack in seemingly healthy people. But half of all heart attacks occur among people who do not have high cholesterol. Also, the classical risk factors of CVD cannot account for all the variation in the incidence of CVD cases [141]. As a result there is a growing interest to identify additional markers of coronary risk. One likely candidate is the C-reactive protein (CRP), although this protein is part of the body's normal response to infection and inflammation. Some of the recent studies have reported elevated CRP levels among those with periodontitis [142–145]. In a study by Ebersole et al., they reported significantly higher levels of CRP among those with adult periodontitis, especially among those having more active sites [146]. The participants of the MI Life Study [143] also reported positive association between elevated levels of CRP (>3 mg/L) and severity of periodontitis. Periodontitis is an inflammatory reaction of the supporting tissues of the teeth like the periodontal ligament, cementum, and alveolar bone to gram-negative anaerobic bacteria. As a response to bacterial endotoxins, the local host inflammatory mediators are activated [94, 147] that in turn initiate localized inflammatory response [148, 149] and finally result in serum antibody response to the bacteria [150, 151]. Bacterial infections may often provide a strong stimulus for a systemic acute phase response that may result in increased production of acute-phase proteins like CRP, macroglobulin, and serum amyloid [152]. In a recent study, it was found that the concentrations of hs-CRP and IL-6 were significantly higher in the sera of patients with periodontitis and periodontal treatment decreased the levels of serum hs-CRP and IL-6 [153]. Elevation of CRP levels among those with periodontitis indicates that periodontitis may also have systemic cytokine mediated effects that may in turn participate in atherogenesis. This may in turn help to explain conditions where dental infections may stimulate systemic inflammatory response, thereby placing “apparently healthy” people at increased risk of cardiovascular disease.

Many works in the literature report familial aggregation of periodontal diseases, but due to different terminology, classification systems, and lack of standardized methods of clinical examination, it is difficult to compare reports directly. Reports of the familial nature of chronic forms of periodontitis are less frequent, although German studies of the familial nature of chronic forms of periodontitis from the early 20th century have been reviewed by [140]. This aggregation within families strongly suggests a genetic predisposition. It must be borne in mind that familial patterns may reflect exposure to common environmental factors within these families.

## 4. Conclusion

It is important to understand the etiological factors and the pathogenesis of periodontal disease to recognize and appreciate the associated risk factors. As periodontal disease is multifactorial, effective disease management requires a clear understanding of all the associated risk factors.
